# Adoption of image surface parameters under moving edge computing in the construction of mountain fire warning method

This article has been retracted.

**DOI:** 10.1371/journal.pone.0232433

**Published:** 2020-05-27

**Authors:** Chen Cheng, Hui Zhou, Xuchao Chai, Yang Li, Danning Wang, Yao Ji, Shichuan Niu, Ying Hou

**Affiliations:** The Second Monitoring and Application Center, CEA, Xi an, China; University College London, UNITED KINGDOM

## Abstract

In order to cope with the problems of high frequency and multiple causes of mountain fires, it is very important to adopt appropriate technologies to monitor and warn mountain fires through a few surface parameters. At the same time, the existing mobile terminal equipment is insufficient in image processing and storage capacity, and the energy consumption is high in the data transmission process, which requires calculation unloading. For this circumstance, first, a hierarchical discriminant analysis algorithm based on image feature extraction is introduced, and the image acquisition software in the mobile edge computing environment in the android system is designed and installed. Based on the remote sensing data, the land surface parameters of mountain fire are obtained, and the application of image recognition optimization algorithm in the mobile edge computing (MEC) environment is realized to solve the problem of transmission delay caused by traditional mobile cloud computing (MCC). Then, according to the forest fire sensitivity index, a forest fire early warning model based on MEC is designed. Finally, the image recognition response time and bandwidth consumption of the algorithm are studied, and the occurrence probability of mountain fire in Muli county, Liangshan prefecture, Sichuan is predicted. The results show that, compared with the MCC architecture, the algorithm presented in this study has shorter recognition and response time to different images in WiFi network environment; compared with MCC, MEC architecture can identify close users and transmit less data, which can effectively reduce the bandwidth pressure of the network. In most areas of Muli county, Liangshan prefecture, the probability of mountain fire is relatively low, the probability of mountain fire caused by non-surface environment is about 8 times that of the surface environment, and the influence of non-surface environment in the period of high incidence of mountain fire is lower than that in the period of low incidence. In conclusion, the surface parameters of MEC can be used to effectively predict the mountain fire and provide preventive measures in time.

## 1. Introduction

China's mountainous area is wide with complex landform and rich resources, including forests, minerals, hydropower, tourism resources, etc., with significant productivity value. But the mountains are covered with vegetation and defoliated leaves. Due to the influence of natural and human activities, fire hazard is extremely easy to occur, which seriously affects the safety of mountain resources and human life and property [1]. At the same time, the occurrence frequency of mountain fires is high, and there is a certain concealment, therefore, there are certain limitations through ground monitoring and early warning. It is very important to adopt appropriate technology to monitor and early warning mountain fires [2]. In order to protect forest resources and people's property, China has adopted a variety of means to monitor and warn mountain fires and achieved certain results [3]. However, there are many factors causing mountain fires, so it is difficult to obtain all of them. Therefore, how to monitor and warn mountain fires through a small number of surface parameters is a hot topic in current research [4].

Image recognition technology has the advantages of high real-time, strong operability, low cost, and large amount of information. Based on the feature extraction and recognition of mountain fire by image and the inversion of surface parameters by remote sensing experimental data, the new method of mountain fire early warning is explored, which has incomparable advantages. However, with the development of image recognition technology, people have higher requirements on the processing power and timeliness of recognition results. The existing mobile phone terminal equipment is insufficient in image processing and storage capacity, and the energy consumption during data transmission is high, so it needs to be unloaded by calculation [5]. Currently, computing tasks are often offloaded to cloud servers to achieve cloud computing via the Internet. However, cloud computing has the defects of high delay, low reliability, and low security [6]. MEC was born to deal with the problems of cloud computing. MEC-based image recognition can be achieved by deploying edge servers; the feature extraction of the image is unloaded to the edge server, and the feature information and projection matrix sent by the cloud server are received instead of sending all data to the cloud server, which can reduce network pressure and transmission delay, and further improve the image recognition effect [7,8].

However, through the investigation of the relevant research at home and abroad, it is found that the research on the use of image recognition technology such as synthetic aperture radar (SAR) imaging for mountain fire early warning and the realization of image recognition algorithm based on moving edge environment has been developed, but the research on the combination of the two is still few. Therefore, this study is based on MEC to identify image surface parameters. Combined with the HDA algorithm, the mountain fire warning model based on MEC is designed to realize effective monitoring and early warning of mountain fire.

## 2. Literature review

### 2.1. Research status of mountain fire early warning model

Matin et al. (2017) calculated a spatially distributed forest fire risk index for Nepal based on a linear model of right weight and grade. The input parameters of the risk assessment model are land cover, temperature, and active fire data, and terrain data based on remote sensor, and the relative risk level is calculated. A total of 18 out of 75 areas are found to be at high risk of forest fires [9]. Pourtaghi et al. (2016) compared the sensitivity map of forest fires based on boosted regression tree (BRT), generalized additive model (GAM), and random forest (RF) data mining model to determine the factors influencing forest fires. The results show that the area under the curve of the forest fire sensitivity map of the three models above ranges from 0.7279 to 0.8770, and the main driving factors for forest fires are annual rainfall, distance to roads, and land use factors [10]. Rui et al. (2018) coupled cellular automata with existing forest fire models to design fire prediction models, and the forest fire spread in the Greater Khingan mountains in May 2006 is tested. The results show that the simulation algorithm of forest fire spread geographic cellular automata is short in time; compared with the real fire data of Landsat Thematic Mapper images, the model has a high temporal and spatial consistency; the average Kappa coefficient is 0.6352 and the average accuracy is 87.89%, which can be used to simulate and predict the spread of forest fires [11]. Qiu et al. (2018) studied a novel flame recognition algorithm in combustion process based on free radical emission spectroscopy, which extracted multiple features from video images and processed the features through time smoothing algorithm to eliminate the false recognition rate. In the time smoothing experiment, the true positive rates of butane flame and forest fire were 0.965 and 0.937, respectively. Experimental results show that the algorithm can accurately identify real fires and determine combustion temperature by CH emission spectrum [12].

### 2.2. The application of MEC in images

Trinh et al. (2018) investigated the potential of MEC to address energy-management related applications on power-constrained limited IoT devices, while also providing low latency processing for visual data generation at high resolution. A novel “unload decision” algorithm is proposed using a face recognition application that is important in disaster event response scenarios. The results show that MEC achieves energy saving through low latency during visual data processing in facial recognition applications, and the performance of this algorithm is better than other algorithms under different user preferences, node mobility, and severe node failure conditions [13]. Hossain et al. (2018) developed an image classification framework using 5G technology. An automatic date fruit classification system is developed in the framework, which combines the deep learning method with the fine-tuned pre-training model, and MEC and cache are used to provide real-time transmission of low-delay and date fruit images [14]. Wu et al. (2018) believed that the enhanced Unikernel can be run as a task in MEC or MFC to effectively support mobile code unloading. To achieve this, the concept of rich-Unikernel is developed to support a variety of applications in a single Unikernel without time-consuming recompilation. Experiments show that compared with traditional virtual machines and containers, Android Unikernel introduces less startup delay, memory consumption, image size, and energy consumption [15].

However, through the investigation of related researches at home and abroad, it is found that the research on mountain fire early warning based on image recognition technology and image recognition algorithm based on moving edge environment has been developed, but there are still few researches on the combination of the two. Based on this, the MEC is used to identify image surface parameters, and an image recognition optimization algorithm is designed under MEC environment. The edge computing environment is combined with the HDA algorithm to give early warning to mountain fires, and the image recognition performance of the algorithm is studied. Taking Muli county, Liangshan prefecture, Sichuan province as an example, the probability of occurrence of mountain fires in this area is predicted.

## 3. Methods

### 3.1. A hierarchical discriminant analysis algorithm for image feature extraction

The HDA algorithm constructs two adjacency matrices for each sample point, the in-class adjacency matrix and the inter-class adjacency matrix. For a given sample xi, it is assumed that its k homogeneous and heterogeneous neighbors sets are respectively $\pi_{k}^{+}\left(x_{i}\right)$ and $\pi_{k}^{-}\left(x_{i}\right)$. The intra-class adjacency matrix F^w^ is expressed as follows.

$$F_{ij}^{w}=\{\begin{array}{l} +1,x_{i}\in \pi_{k}^{+}\left(x_{j}\right)\;or\;x_{j}\in \pi_{k}^{+}\left(x_{i}\right)\\ \begin{array}{ll} 0 & otherwise \end{array} \end{array}$$ (1)

The class adjacency matrix F^h^ is expressed as follows.

$$F_{ij}^{h}=\{\begin{array}{l} +1,x_{i}\in \pi_{k}^{-}\left(x_{j}\right)\;or\;x_{j}\in \pi_{k}^{-}\left(x_{i}\right)\\ \begin{array}{ll} 0 & otherwise \end{array} \end{array}$$ (2)

The sum of the distance within the class after projection can be expressed as follows.

$$\begin{array}{ll} \Phi \left(P_{1}\right) & =\sum_{x_{i}\in \pi_{k}^{+}\left(x_{j}\right)}\sum_{x_{j}\in \pi_{k}^{+}\left(x_{i}\right)}{\left\|P_{1}^{T}x_{i}-P_{1}^{T}x_{j}\right\|}^{2}F_{ij}^{w}\\ & =2P_{1}^{T}X\left(D^{w}-F^{w}\right)X^{T}P_{1} \end{array}$$ (3)

Among them, D^w^ represents a diagonal matrix, that is, the sum of the columns whose diagonal elements are F^w^. Firstly, the sum of distances within the class is optimized. Samples of the same category should meet in the projection space, that is, the smaller the distance between samples is, the better. Therefore, the objective function can be expressed as follows.

$$\left\{ \begin{array}{l} \underset{P_{1}}{\text{min}}tr\{P_{1}^{T}XSX^{T}P_{1}\}\\ s.t.P_{1}^{T}P_{1}=1 \end{array}\right.$$ (4)

Similar to the representation of the sum of the distance within the class, the sum of the distance between the classes after projection can be expressed as follows.

$$\begin{array}{ll} \Psi \left(P\right) & =\sum_{x_{i}\in \pi_{k}^{-}\left(x_{j}\right)}\sum_{x_{j}\in \pi_{k}^{-}\left(x_{i}\right)}{\left\|P^{T}x_{i}-P^{T}x_{j}\right\|}^{2}\\ & =2P^{T}X\left(D^{h}-F^{h}\right)X^{T}P \end{array}$$ (5)

Among them, D^h^ represents a diagonal matrix, that is, the sum of the columns whose entries on the diagonal are F^h^. Then, the second step is to optimize the sum of distances between classes. In the projection space, the greater the distance between sample points of different classes, the better. Therefore, when the sum of distances between classes is optimized, it should be maximized. The objective equation is as follows.

$$\left\{ \begin{array}{l} \underset{P}{\text{min}}tr\{P^{T}X_{new}MX_{{}^{new}}^{T}P\}\\ s.t.P^{T}P=1 \end{array}\right.$$ (6)

Since S and M are real symmetric matrices, the optimization Eqs 4 and 6 are transformed into the eigendecomposition problem of matrices XSX^T^ and XMX^T^. The two projection matrices P are composed of the eigenvectors of XSX^T^ and XMX^T^, that is, P_1_ and P are in the form of *P* = [*P*_1_,…, *P*_*r*_]. Therefore, any sample point xi can be expressed as $v_{i}=P^{T}x_{i}$.

The specific steps of the algorithm are as follows.

Input: training sample set ${\left\{\left(x_{i},y_{i}\right)\right\}}_{i=1}^{N}$, the subspace dimension of the reduced dimension is r.

Output: projection matrix P.

1. The intra-class adjacency matrix graph F^w^ and inter-class adjacency matrix graph F^h^ are constructed.

2. The matrix XSX^T^ is decomposed to minimize the sum of distances within the class, among them *S* = *D*^*w*^ − *F*^*w*^. The eigenvalue of the matrix after the fearure decomposition is *λ*_*i*_, *i* = 1,…, *d*, and its corresponding eigenvectors are arranged in ascending order, there is *λ*_1_ ≤ *λ*_2_ ≤ … *λ*_*d*_.

3. The first r minimum eigenvalues are selected to form the eigenvector matrix *P* = [*P*_1_,…, *P*_*r*_].

4. The new training sample is calculated as the new input.

5. The sum of the distances between classes is maximized by decomposing the matrix XMX^T^, among them, *S* = *D*^*h*^ − *F*^*h*^. The eigenvalue of the matrix after the feature decomposition is *λ*_*i*_, *i* = 1,…, *d*, and its corresponding eigenvectors are arranged in decending order, there is *λ*_1_ ≥ *λ*_2_ ≥ … *λ*_*d*_.

6. The first r maximum eigenvalues are selected to form the eigenvector matrix *P* = [*P*_1_,…, *P*_*r*_], returning to projection matrix P.

### 3.2. The design of mobile image acquisition software

The developed image capture software is deployed on Android phone. Android applications are developed through Android SDK using Java programming language. Each application can run on its own independent virtual machine. This virtual machine supports JNI and has an Android NDK, so programs can be written using third-party C/C++ libraries. OpenCV consists of a series of C functions and C++ classes. It is an open source, cross-platform computer vision library based on BSD license, which can realize algorithms in image processing and other aspects. Therefore, the OpenCV can be used for image recognition in android system.

Android application development is written in the Java programming language, so it needs to configure the Java development environment on Windows. The appropriate JDK environment variables are downloaded and configured and Android Studio is installed. Then the OpenCV4Android SDK is updated and it is configured into the android system. The android.mk file and code are modified so that it can run application opencv-like programs without the need for OpenCV Manager.

In order to collect, transmit, and process images and display recognition results, the developed software needs to have the functions of image acquisition and upload, image grayscale, and displaying recognition results, as shown in Table 1.

**Table 1:** Functions of the software.

Image acquisition and upload function	The image is selected from the album or taken and uploaded to the edge server, and the socket can be used for upload.
Image graying function	Before sending the image, OpenCV is used for grayscale processing to reduce the transmission of redundant information.
Displaying recognition result function	The image recognition results can be obtained intuitively and the response time can be returned.

Image upload function. In the application's MainActivity, the "taking image" and "album selecting" buttons are set. After selecting image, the thumbnail of the selected image is displayed on the main page, and the recognition result and response time of the image are displayed on the page.

Image grayscale function. After selecting the image, OpenCV is used to convert the color image to the gray image for histogram equalization. Then the classifier is used to detect an area in the image. OpenCV stores the classifier information in an XML file in the asset folder under the Java project directory, and this file can be written to the specified path when the application is installed. The detected information is stored in the face with data type Rect, and the image is clipped and grayed according to the location information. Finally, the network is connected, the image is uploaded to the edge server via socket, and the result is returned.

### 3.3. Image recognition and optimization algorithm under MEC environment

With the explosive growth of mobile traffic and the combination of 5G and Internet of things, the use of MCC architecture leads to core network congestion and network transmission delay. Today, applications such as virtual and augmented reality require less latency, leading to the emergence of mobile edge computing architectures. Mobile edge computing uses the edge of the user's mobile terminal (data source), that is, the edge server on the base station, to complete the computing task, and performs edge big data processing in a distributed way. Mobile edge computing is more suitable for real-time data analysis and intelligent processing, and more efficient than simple MCC. MEC aims to provide IT service environments and cloud computing capabilities on the edge of mobile networks. The mobile edge computing platform increases the computing responsibilities of the edge server, allowing the edge server to compute and service, thereby reducing network latency and bandwidth consumption at the user end.

MEC is to solve the transmission delay problem caused by traditional MCC. The edge servers are used to provide compute storage resources for applications, and the edge of big data processing is carried out in a distributed way. MEC is better for real-time data analysis than MCC. Its computing architecture consists of the user, the edge server, and the cloud server, as shown in Fig 1.

**Fig 1:** MEC architecture.

In image recognition, it is very important to get the response time of the recognition result. However, the processing power of the mobile phone can't meet the requirement of fast computing to obtain the results, while the processing power of the cloud server is strong, but its long distance will slow the response time. Therefore, mobile terminal computing can be offloaded to the edge server for image recognition processing, which can relieve the pressure of mobile phone processing big data. At the same time, edge servers are closer than cloud servers, with faster recognition speed, and less response time.

The image recognition and optimization algorithm architecture under MEC Environment is shown in Fig 2. MEC infrastructure is divided into mobile devices, edge servers, and cloud servers. Images are collected by mobile devices and uploaded to the edge server. Then the edge server is trained by the cloud server to obtain the projection matrix, to extract the discriminant information. After comparison with the feature information base, the recognition result is obtained and returned to the mobile device. Meanwhile, the image feature information will be sent to the cloud server as a new training sample. The server obtains the projection matrix and feature information through the training sample image, sends it to the edge server, and receives the new image features returned by the edge server for training again.

**Fig 2:** Application architecture of image recognition optimization algorithm under MEC environment.

#### a. Users

Mobile devices only serve as the front end of image acquisition programs because of the lack of computing, processing and image storage capabilities of mobile phones. The images to be identified can be collected on the mobile phone and selected through shooting or album. After the selected image is grayed, it is uploaded to the edge server through the base station, and the recognition result of the image is received at the mobile phone terminal. Since grayscale images are easy to process, users can greyscale color images through OpenCV and then use socket to upload them to the edge server.

#### b. The edge servers

The base station server is taken as the edge server. Its computing and storage capacity is good, but its storage capacity is insufficient. Therefore, image information in the database needs to be stored in the cloud server. The edge server can receive the image feature information and projection matrix of the storage cloud server for image recognition. The image recognition process of edge server is as follows.

The edge server receives the image sent by the mobile phone terminal, extracts the feature information according to the projection matrix, and returns the image recognition result to the user. The training model is also received from the cloud server. In this study, the computer is selected as the edge server, and the edge server has a dual role. One is to receive the image feature information and projection matrix sent by the cloud server; the other is to receive images sent by mobile terminals, the image information to be identified is extracted through the projection matrix and compared with the features in the database, and the value with the highest similarity is returned to the user as the recognition result.

#### c. The cloud servers

The cloud server is rich in resources and has strong computing power, which can be applied to the existing cloud server for processing. In the cloud server, it mainly stores the image information of the database, extracts the key features of the trained image information, and sends the image feature information and projection matrix to the edge server.

In this study, TenCent cloud is selected as the cloud server, and HDA algorithm is applied to train the image and obtain the projection matrix P. Then, the image feature information is extracted according to the projection matrix and sent to the edge server to identify the image in the form of image name and key value pairs of feature information. Meanwhile, the image feature information recognized by the edge server is sent to the cloud server. As a new training sample, a new projection matrix and feature information base are obtained and sent to the edge server again to improve the image recognition accuracy.

Fig 3 shows the identification flow of the system.

**Fig 3:** The image recognition process under MEC environment.

### 3.4. Construction of the experimental environment

In this experiment, two network connection modes, WiFi and mobile cellular network, are adopted to support the advantages of MEC architecture from response time and data transmission volume.

In order to implement a MEC environment, it is necessary to deploy virtualized servers in multiple locations on the edge of the mobile network. Experimental simulation is carried out by self-built base station, which is built based on Open Air Interface, including rf signal generator, base station server A, and base station server B. The rf signal generator is USRP-B210. Base station server A is a computer loaded with Ubuntu, Intel i7 processor and 16GB of memory. The RF signal generator is linked to base station A via USB3.0. Base station server B is a computer loaded with Ubuntu, Intel i5 processor and 4 GB of memory. Base station server A and base station server B are connected via LAN. The MEC server consists of two computers.

### 3.5. The mountain fires early warning model based on MEC

Forewarning of forest fires requires certain threshold standards. According to different conditions in different areas, there are many forest fire risk indexes. The main factors that determine forest fire risk include the moisture content of fuel and weather conditions, in which the moisture content of fuel is affected by vegetation growth, soil moisture, temperature, and other factors. At present, the forest fire risk index of early warning mountain fire is widely used, including fire weather index (FWI) [16], FSI [17] and fire potential index (FPI) [18]. Forest fire index is usually evaluated by meteorological information and optical image information, and it has certain limitations in the case of complex terrain and meteorology. The input parameters of forest fire risk index can be obtained by sensor measurement, historical data, or remote sensing data.

FSI combines remote sensing data with meteorological conditions, and introduces into it the physical quantity describing the ignition energy of the fuel, namely the ignition energy, which refers to the amount of energy required to raise the fuel from the current temperature to the ignition point. The forest fire risk index refers to the energy needed to ignite the object and the ignition energy can represent the inflammability of the combustible, thus achieving the forewarning effect of mountain fire. The calculation equation of FSI is as follows.

$$FSI=\left[\frac{\left(Q_{igavg}-Q_{ig}\right)}{Q_{igavg}}\right]\times 100$$ (7)

In Eq 7, *Q*_*ig*_ represents ignition energy; *Q*_*igavg*_ is the average ignition energy. If FSI is positive, it means that the average state of fire risk ratio in the region is higher, and vice versa. The higher the FSI value, the higher the probability of fire. Due to the large time series, the FSI values of the live fuel (the fuel moisture content is above 30%) and the dead fuel (the fuel moisture content is below 30%) are not the same, so they need to be calculated separately. After weight analysis, the comprehensive FSI value is finally obtained. The calculation equation is as follows.

$$FSI=W_{L}\cdot FSI_{L}+W_{D}\cdot FSI_{D}$$ (8)

In Eq 8, W_L_ and W_D_ represent the weights of live and dead combustible in the whole region. In Sichuan, W_L_ is 0.22, and W_D_ is 0.78.

Through the above analysis of forest fire risk index, it can be concluded that FSI can accurately predict the probability of forest fire, that is, the image feature information of MEC is input into the warning model to show the probability of mountain fire.

The MEC is first used to invert soil water content in vegetation covered areas. Combining moisture content parameter Moss and FSI model to calculate the probability of forest fire, it can be expressed by Eq 9.

$$\left\{ \begin{array}{l} FSI>\gamma \left(\gamma >10\right)\\ Moss<\tau \left(\tau >0\right) \end{array}\right.$$ (9)

For the studied area of Muli county, Liangshan prefecture, the distribution of soil water content is adjusted according to the distribution of soil water content. The range of τ is defined between 10%-20%. The expression of the prediction model is obtained as Eq 10.

$$FSI_{new}=\left\{ \begin{array}{l} \frac{\left(2053.65+1.7T_{f}\right)Bio_{v}-\left(1561.751-4.187T_{f}\right)M_{v}}{3073.65Bio_{v}}\times 100\left[M_{v}>0.2\right]\\ \frac{\left(2.73+1.7T_{f}\right)Bio_{v}-\left(1561.751-4.187T_{f}\right)M_{v}}{1022.73Bio_{v}}\times 100\left[M_{v}\leq 0.2\right]\\ M_{s}\leq 0.2\left[High\right]\\ 0.2<M_{s}\leq 0.4\left[Middle\right]\\ M_{s}>0.4\left[Low\right] \end{array}\right.$$ (10)

In Eq 10, T_f_ represents the surface temperature; M_v_ represents the water content of vegetation; Bio_v_ is the biomass of vegetation; M_s_ is the soil moisture content. Soil moisture content is a threshold value, which can be used together with FSI to judge the probability of hill fires. When the FSI value is high and the soil moisture content is low, the probability of hill fires is high, and vice versa.

### 3.6. Data set

When testing the performance of the image recognition optimization algorithm in the MEC environment, the data set used is UMIST [19]. The sample size of this dataset is 574, the dimension is 1024, the number of categories is 20, and the original size of each image is 112×92 pixels.

Radarsat-2 satellite data is used for the prediction of wildfires [20]. Radarsat-2 images obtained from Muli county, Liangshan prefecture on April 21, 2018 and September 26, 2018 are used. Detailed parameter information is shown in Table 2. Along with the satellite image, the field measurements are carried out to obtain the soil moisture content and vegetation parameters in the area.

**Table 2:** Related parameters of Radarsat-2 image in Muli county, Liangshan prefecture.

Product types	Beam pattern	Range of incident angles	Polarization mode	Resolution ratio	Image size
Single look complex (SLC)	Fine full polarization (FQ24)	20°-41°	HH/VV/HV/VH	5.2×7.6 m	25×25 km

## 4. Results

### 4.1. Performance comparison of hierarchical discriminant analysis algorithm

In order to verify the performance of the hierarchical discriminant analysis algorithm, the hierarchical discriminant analysis is compared with other representative feature extraction algorithms MFA [21], LDNE [22], and DAG-DNE [23]. In the experimental process, all data are firstly reduced to 100 dimensions by principal component analysis algorithm, which can reduce the complexity of data calculation and effectively remove noise. The experimental data sets include Yale data set [24], UMIST data set, and ORL data set [25].

Table 3 shows the comparison of the average recognition accuracy of four different algorithms in the parameter K value of different number of neighbors. In the case of three data sets with different number of neighbors, HDA has higher recognition accuracy than other three algorithms, and the recognition accuracy is up to 98% when the number of neighbors in ORL data set is 3. In the Yale data set, the hierarchical optimization of HDA presents better recognition results than the simultaneous optimization of LDNE, MFA, and DAG-DNE, which exceeds 6.7% of the second-best algorithm. In the UMIST data set, when the number of neighbors is 1, the recognition accuracy of HDA is nearly 18% higher than that of LDNE algorithm. In these data sets, hierarchical discriminant analysis presents better results, possibly because the difference between the sum of intra-class distances and the sum of inter-class distances of these data sets is too large, and the local feature structure of the original data is better retained by hierarchical optimization. From the experimental data, it is found that the hierarchical discriminant analysis algorithm optimizes the sum of intra-class distance and inter-class distance separately by learning the advantages of the layered strategy of deep learning, which effectively improves the classification performance of the algorithm. And it can be found from the data that the HDA algorithm can achieve the optimal recognition effect when the number of features is obtained.

**Table 3:** The accuracy of each algorithm in different number of neighbors in different data sets.

Data sets	Yale			UMIST			ORL		
	K = 1	K = 3	K = 5	K = 1	K = 3	K = 5	K = 1	K = 3	K = 5
LDNE	0.47	0.45	0.47	0.96	0.94	0.94	0.93	0.92	0.91
MFA	0.67	0.83	0.78	0.95	0.96	0.98	0.93	0.94	0.94
DAG-DNE	0.69	0.80	0.76	0.96	0.96	0.96	0.95	0.96	0.94
HDA	0.78	0.87	0.80	0.97	0.97	0.97	0.94	0.98	0.96

### 4.2. Image recognition optimization algorithm performance under MEC environment

In order to verify the superiority of MEC over MCC and the optimization performance of layered discriminant analysis algorithm for MEC, in this study, the proposed HDA algorithm (MECHDA) in the MEC environment is compared with the HDA (MCCHDA) in MCC, the general feature extraction algorithm (MEC Simple) in MEC, and the general feature extraction algorithm (MCC Simple) in MCC. The bandwidth and response time of different algorithms are investigated, and two network conditions of WiFi and mobile data network are simulated.

MCC Simple is the MCC framework. The user directly transmits the original image to the cloud server, extracts the features through the PCA algorithm, and then directly recognizes them. The user receives the recognition results from the cloud server. Compared with MCC Simple, MCCHDA applies layered discriminant analysis to extract feature information and learn projection matrix P in cloud server. MEC Simple uses the mobile edge computing architecture to transfer the original image to the edge server and complete the image recognition. The MECHDA framework combines the MEC with the layered discriminant analysis algorithm, and sends the feature information of the image database to the edge server, and the identification is completed in the edge server.

Figs 4 and 5 respectively show the response time of different images of different system architectures under the two network simulation conditions, and images of different sizes are numbered 1–5. As shown in the figure, the response time of image recognition is more than twice different between WiFi and mobile data network. Among them, the image recognition response time under WiFi network is less than 800 ms, and the image recognition response time under mobile data network is between 1000–3000 ms. MECHDA has the fastest response time for different images. It can be concluded from this that MEC is closer to the user than MCC, and the image recognition response time is faster. Compared with MCC, MEC architecture can make recognition close to the user and accelerate the response time of image recognition.

**Fig 4:** The response time of each architecture under the mobile data network.

**Fig 5:** Response times for each architecture under WiFi.

Table 4 shows the bandwidth consumption under different architectures. In the MCC framework, what is transmitted is the size of the whole image, and only the feature information of the image is transmitted. MECHDA transmits 1KB of image feature information, and MEC combined with HDA algorithm transmits less data, which can effectively reduce the network bandwidth pressure.

**Table 4:** Bandwidth usage for different architectures.

Bandwidth usage	MCCSimple	MCCHDA	MECSimple	MECHDA
Image 1	612.43 KB	541.50 KB	56.79 KB	1 KB
Image 2	1031.88 KB	970.08 KB	20.93 KB	1 KB
Image 3	1326.31 KB	1249.78 KB	23.92 KB	1 KB
Image 4	1329.08 KB	1247.34 KB	37.89 KB	1 KB
Image 5	2706.89 KB	2640.38 KB	54.23 KB	1 KB

### 4.3. Mountain fire prediction results

In this study, images of the low occurrence period (September 2018) and the high occurrence period (April 2018) of wildfires are selected. According to the FSI and FSI_new_, the fire risk level is divided into 6 levels, 1 is the lowest, 6 is the highest, and 2 is the higher fire risk area. After FSI_new_ corrects the soil moisture data, when the soil moisture content is less than 20%, the surface environment is more likely to cause forest fires. When the soil moisture content is higher than 20%, the factors influencing the non-surface environment are greater. Among them, the surface environmental factors include drought, ground temperature, etc., while the non-surface environment mainly includes man-made activities and lightning weather activities.

Table 5 shows the distribution and possible factors of mountain fires in Muli county, Liangshan prefecture during the low and high season. The proportion of fire risk in Muli county of Liangshan prefecture below 2 is more than 90%, indicating that the probability of mountain fires in most areas of the region is low and relatively safe. In the areas with low occurrence of wildfires and high fire risk, the probability of non-surface environment causing wildfires is 86%, while in the areas with high occurrence of wildfires, the probability of non-surface environment causing wildfires is 82%, which shows that the probability of mountain fires caused by the non-surface environment in Muli county, Liangshan prefecture is about 8 times that of the surface environment. At the same time, it shows that the influence of the non-surface environment in the high season of mountain fires is lower than that in the low season, indicating that the climate environment in this region is dry and the weather conditions such as thunder and lightning are less in the high season, and mountain fires are mainly caused by the surface environment at this time.

**Table 5:** Analysis on distribution and possible factors of mountain fires in Muli county, Liangshan prefecture during low and high occurrence periods.

Levels	Surface environmental factors				Non-surface environmental factors			
	Pixel data		Proportion		Pixel data		Proportion	
	Low occurrence period	High occurrence period	Low occurrence period	High occurrence period	Low occurrence period	High occurrence period	Low occurrence period	High occurrence period
1	288764	221043	0.9550	0.9371	0	0	0	0
2	9264	8992	0.0313	0.0381	0	0	0	0
3	2901	3147	0.0092	0.0133	6257	5679	0.1809	0.1836
4	1142	1760	0.0036	0.0075	7642	6771	0.2209	0.2190
5	251	723	0.0008	0.0031	8318	7146	0.2404	0.2311
6	41	204	0.0001	0.0009	12379	11328	0.3578	0.3663

## 5. Discussion

The purpose of this study is to predict mountain fires. Based on MEC, stratified discriminant analysis algorithm is implemented to extract surface parameter characteristics of mountain fire. Then a forest fire early warning model based on MEC is designed, the performance of the algorithm is studied, and the occurrence probability of forest fire in Muli county, Liangshan prefecture, Sichuan is predicted. The algorithm described in this study has a high recognition accuracy. Compared with the MCC architecture, when MEC is combined with the layered discriminant analysis algorithm, the response time of the recognition image is faster and the amount of data transmitted is smaller, which conforms to the expected effect in the early stage of model design. Because compared with other algorithms, under the same recognition rate, HAD requires less feature information and high recognition rate, so the corresponding computation is less and the processing and recognition of the image takes less time. At the same time, because of the deployment of hierarchical discriminant analysis algorithm, the accuracy of image recognition is also high. Liu and Zhao (2019) proposed a hierarchical feature extraction algorithm based on discriminant analysis, which decomposed highly complex feature extraction problems into smaller problems without determining the optimal feature subset size. On different types of data sets and typical classifiers, the effectiveness and efficiency of the algorithm show good performance [26]. When the occurrence probability of mountain fire in Muli county of Liangshan prefecture is predicted, it is found that the probability of forest fire in most areas of the region is low, and the probability of forest fire caused by non-surface environment is high, and the influence of non-surface environment in the period of high incidence of forest fire is lower than that in the period of low incidence. Pandeyd and Ghosh (2018) used remote fire risk model generation to map fire risk area sensing and GIS technology. Forest fire risk model is generated by AHP method. Each model assigns a subjective weight to the category according to the sensitivity to fire. The three categories of forest fire risk are obtained from high to low. The results show that the generated forest fire risk model is highly consistent with the actual fire location [27]. The fire prevention measures can be carried out targeted in the Liangshan prefecture Muli county area according to the mountain fire occurrence probability, such as paying attention to prevent in the lightning season or when human activities are frequent (burning straw, sacrifice, etc.).

## 6. Conclusion

In this study, ground surface parameters of image are identified based on MEC. The image capture software under MEC environment is designed and installed in android system, the images to be recognized are collected, the image recognition optimization algorithm in the MEC environment is designed, and they are combined with the HDA algorithm. According to the FSI, the mountain fire warning model based on MEC is designed. The performance of the algorithm is compared and the probability of mountain fire occurrence in Muli county, Liangshan prefecture, Sichuan province is predicted. Compared with the MCC architecture, the algorithm described in this study has a shorter response time for recognition of different images in the WiFi network environment and a smaller amount of transmitted data, which can effectively reduce the network bandwidth pressure. The probability of mountain fire caused by non-surface environment in Muli county, Liangshan prefecture is about 8 times higher than that of surface environment. This study can effectively predict mountain fires based on the surface parameters of MEC images and provide timely preventive measures. However, image recognition based on moving edge environment is shallow learning, which is still insufficient for image recognition under deep learning. This kind of research method can also be used in the study of spatial change of foundation settlement and water eutrophication [28]. Therefore, in the follow-up research work, it needs to focus on in-depth learning, so that it can be better applied to the actual situation.

## Supporting information

S1 Data (XLSX)

## References

[1] LiJ., YanB., ZhangM., et al (2019) “Long-range raman distributed fiber temperature sensor with early warning model for fire detection and prevention”, *IEEE Sensors Journal*, 19(10), pp.3711–3717.

[2] LindenmayerD. B., SatoC. (2018) “Hidden collapse is driven by fire and logging in a socioecological forest ecosystem”, *Proceedings of the National Academy of Sciences*, 115(20), pp.5181–5186.10.1073/pnas.1721738115PMC596030729712832

[3] DaviesK. W., BatesJ. D., HuletA. (2017) “Attempting to restore mountain big sagebrush (Artemisia tridentata ssp. vaseyana) four years after fire”, *Restoration Ecology*, 25(5), pp.717–722.

[4] BoerM. M., NolanR. H., De DiosV. R., et al (2017) “Changing weather extremes call for early warning of potential for catastrophic fire”, *Earth's Future*, 5(12), pp.1196–1202.

[5] AbrahimA. R., RahimM. S. M., SulongG. B. (2019) “Splicing image forgery identification based on artificial neural network approach and texture features”, *Cluster Computing*, 22(1), pp.647–660.

[6] QinC., QianZ., FengG., et al (2019) “Special issue on real-time image watermarking and forensics in cloud computing”, *Journal of Real-Time Image Processing*, 16(3), pp.559–563.

[7] HaoY., ChenM., HuL., et al (2018) “Energy efficient task caching and offloading for mobile edge computing”, *IEEE Access*, 6, pp.11365–11373.

[8] HsiehH. C., LeeC. S., ChenJ. L. (2018) “Mobile edge computing platform with container-based virtualization technology for IoT applications”, *Wireless Personal Communications*, 102(1), pp.527–542.

[9] MatinM. A., ChitaleV. S., MurthyM. S., et al (2017) “Understanding forest fire patterns and risk in Nepal using remote sensing, geographic information system and historical fire data”, *International journal of wildland fire*, 26(4), pp.276–286.

[10] PourtaghiZ. S., PourghasemiH. R., AretanoR., et al (2016) “Investigation of general indicators influencing on forest fire and its susceptibility modeling using different data mining techniques”, *Ecological indicators*, 64, pp.72–84.

[11] RuiX., HuiS., YuX., et al (2018) “Forest fire spread simulation algorithm based on cellular automata”, *Natural hazards*, 91(1), pp.309–319.

[12] QiuX., XiT., SunD., et al (2018) “Fire detection algorithm combined with image processing and flame emission spectroscopy”, *Fire technology*, 54(5), pp.1249–1263.

[13] TrinhH., CalyamP., ChemodanovD., et al (2018) “Energy-aware mobile edge computing and routing for low-latency visual data processing”, *IEEE Transactions on Multimedia*, 20(10), pp.2562–2577.

[14] HossainM. S., MuhammadG., AminS. U. (2018) “Improving consumer satisfaction in smart cities using edge computing and caching: A case study of date fruits classification”, *Future Generation Computer Systems*, 88, pp.333–341.

[15] WuS., MeiC., JinH., WangD. (2018) “Android unikernel: Gearing mobile code offloading towards edge computing”, *Future Generation Computer Systems*, 86, pp.694–703.

[16] VarelaV., SfetsosA., VlachogiannisD., et al (2018) “Fire Weather Index (FWI) classification for fire danger assessment applied in Greece”, *Tethys*, 15, pp.31–40.

[17] CollinsL., GriffioenP., NewellG., et al (2018) “The utility of Random Forests for wildfire severity mapping”, *Remote Sensing of Environment*, 216, pp.374–384.

[18] AdelabuS. A., AdepojuK. A., MofokengO. D. (2020) “Estimation of fire potential index in mountainous protected region using remote sensing”, *Geocarto International*, 35(1), pp.29–46.

[19] GrahamDaniel B., and AllinsonNigel M. "Characterising virtual eigensignatures for general purpose face recognition" Face Recognition. Springer, Berlin, Heidelberg, 1998 446–456.

[20] MahdianpariM., SalehiB., MohammadimaneshF., MotaghM. (2017) “Random forest wetland classification using ALOS-2 L-band, RADARSAT-2 C-band, and TerraSAR-X imagery”, *ISPRS Journal of Photogrammetry and Remote Sensing*, 130, pp.13–31.

[21] ZhangJ., TengY. F., ChenW. (2019) “Support vector regression with modified firefly algorithm for stock price forecasting”, *Applied Intelligence*, 49(5), pp.1658–1674.

[22] DingC., WangS. (2019) “Appropriate points choosing for subspace learning over image classification”, *The Journal of Supercomputing*, 75(2), pp.688–703.

[23] ZhaoG., ZhouZ. (2019) “Efficient Linear Feature Extraction Based on Large Margin Nearest Neighbor”, *IEEE Access*, 7, pp.78616–78624.

[24] AbuzneidM. A., MahmoodA. (2018) “Enhanced human face recognition using LBPH descriptor, multi-KNN, and back-propagation neural network”, *IEEE Access*, 6, pp.20641–20651.

[25] LinW. A. N. G., Fang-JuanD. E. N. G. (2018) “Improved Weighted Sparse Representation Algorithm for Face Recognition”, *Computer Systems & Applications*, 27(6), pp.134–139.

[26] LiuX., ZhaoH. (2019) “Hierarchical feature extraction based on discriminant analysis”, *Applied Intelligence*, 49(7), pp.2780–2792.

[27] PandeyK., GhoshS. K. (2018) “Modelling of Parameters for Forest Fire Risk Zone Ma*pping**”*, *ISPRS-International Archives of the Photogrammetry*, *Remote Sensing and Spatial Information Sciences*, XLII, 5, pp.299–304.

[28] YangH. Q., ZhangL., & LiD. Q. (2018). Efficient method for probabilistic estimation of spatially varied hydraulic properties in a soil slope based on field responses: A Bayesian approach. *Computers and Geotechnics*, 102, pp.262–272.

